The article "Effect of harvest season on the nutritional value of bee pollen protein" was retracted in 2022. Reasons: compromised peer review; a conflict of interest; concerns about the authorship.

# Effect of harvest season on the nutritional value of bee pollen protein

**DOI:** 10.1371/journal.pone.0241393

**Published:** 2020-12-28

**Authors:** Saad N. Al-Kahtani, El-Kazafy Taha, Khalid Ali Khan, Mohammad Javed Ansari, Soha A. Farag, Dalia M. B. Shawer, El-Said Mohamed Elnabawy

**Affiliations:** 1 Arid Land Agriculture Department, College of Agricultural Sciences & Foods, King Faisal University, Al-Ahsa, Saudi Arabia; 2 Faculty of Agriculture, Economic Entomology Department, Kafrelsheikh University, Kafrelsheikh, Egypt; 3 Research Center for Advanced Materials Science (RCAMS), King Khalid University, Abha, Saudi Arabia; 4 Faculty of Science, Unit of Bee Research and Honey Production, King Khalid University, Abha, Saudi Arabia; 5 Faculty of Science, Biology Department, King Khalid University, Abha, Saudi Arabia; 6 Department of Botany, Hindu College Moradabad, Moradabad, Uttar Pradesh, India; 7 Faculty of Agriculture, Department of Animal and Poultry Production, University of Tanta, Tanta, Egypt; Harran University, TURKEY

## Abstract

Bee pollen is a natural product that has valuable nutritional and medicinal characteristics and has recently garnered increasing attention in the food industry due to its nutritive value. Here, we harvested pollen loads from the Al-Ahsa oasis in eastern Saudi Arabia during spring, summer, autumn, and winter in 2018/2019 to compare the nutritional value of bee pollen protein with the amino acid requirements of honeybees and adult humans. Based on the nutritional value of bee pollen protein, the optimal season for harvesting bee pollen was determined. The composition of the bee pollen showed the highest contents of crude protein, total amino acids, leucine, glutamic acid, valine, isoleucine, threonine, and glycine in samples collected in spring. The highest contents of lysine, phenylalanine, threonine, tryptophan, arginine, tyrosine, and cysteine were observed in samples collected in winter. The highest contents of histidine, methionine, and serine were in samples collected in autumn. Moreover, the highest levels of aspartic acid, proline, and alanine were in samples collected in summer. Leucine, valine, lysine, histidine, threonine, and phenylalanine (except in autumn bee pollen) contents in pollen from all four seasons were above the requirements of honeybees. Leucine, valine, histidine, isoleucine (except in autumn bee pollen), lysine (except in spring and summer bee pollen), and threonine (except in winter and spring bee pollen) in all tested samples were above the requirements of adult humans. In comparison with the minimal amino acid requirements of adult humans and honeybees, the 1^st^ limiting amino acid in bee pollen collected during the different seasons was methionine. Bee pollen collected during spring (March–May) and winter (December–February) can be considered a nutritive food source for adult humans and honeybees.

The article "Effect of harvest season on the nutritional value of bee pollen protein" was retracted in 2022. Reasons: compromised peer review; a conflict of interest; concerns about the authorship.

## Introduction

Pollen and nectar are natural foods of honeybees. Bee pollen is the principal nutrient resource for adult and larval bees, which have nutritive requirements for development [1–3]. In addition, bee pollen has been used as a supplementary food in human health [4–7] and poultry diets [8–10].

The physicochemical and nutritional characteristics of bee pollen vary greatly according to its botanical and geographical origins [11–15]. Bee pollen consists of nutritive and bioactive compounds [2,16,17]. The protein concentration in bee pollen varies between 10% and 40% and is affected by botanical origin [2,3,11,12,14,18].

Approximately 16 amino acids are found in bee pollen [11,18–22]. Ten amino acids (leucine, valine, lysine, isoleucine, histidine, threonine, tyrosine, phenylalanine, tryptophan, and methionine) called essential amino acids (EAAs) which cannot be synthesized by the human body [23], and they must be included in the human diet. Moreover, the EAAs for honeybees are leucine, lysine, isoleucine, histidine, arginine, valine threonine, phenylalanine, tryptophan, and methionine [24]. Bee pollen was recorded as a rich source of EAAs [12,18,25,26]. The proportion of EAAs in bee pollen ranged between 34.59% and 48.49% [18–21]. The prevalent amino acids in bee pollen are glycine, aspartic acid, glutamic acid, alanine, leucine, valine, lysine, serine, and isoleucine [12,18,21,27–29].

Alfalfa (*Medicago sativa* L.), date palm (*Phoenix dactylifera* L.), rapeseed (*Brassica napus* L.), summer squash (*Cucurbita pepo* Thunb), and sunflower (*Helianthus annuus* L.) are the major pollen floral resources for honeybees in the Al-Ahsa oasis, Saudi Arabia, and they contributed approximately 93.97% to 94.76% of the yearly collected bee pollen [11,30]. Significant variations in the amino acid composition of bee pollen from these sources have been found by Taha et al. [18]. Unfortunately, the collection of separate pollen loads from these major sources is difficult and requires a long time. Therefore, a seasonal study on the amino acid composition of bee pollen led to the identification of the optimal period for harvesting pollen. However, seasonal variations in the amount of collected bee pollen and its nutrient content have been found [13]. We aimed to estimate the nutritive value and amino acid contents in bee pollen and compared them to the requirements of honeybees (*A*. *mellifera* L.) and adult humans; additionally, the optimal season for harvesting bee pollen with the best nutritive value in terms of protein was determined.

The article "Effect of harvest season on the nutritional value of bee pollen protein" was retracted in 2022. Reasons: compromised peer review; a conflict of interest; concerns about the authorship.

## Materials and methods

### Experimental sites

Five divergent apiaries in the Al-Ahsa oasis (25°25′46″N, 49°37′19″E; 121 m above sea level) in eastern Saudi Arabia were selected for bee pollen collection. Temperature, relative humidity, rainfall rate, and soil characteristics for all five apiaries were relatively similar while, the major pollen and nectar plants were totally different at locations where the five apiaries were present (Table 1).

**Table 1:** Major pollen and nectar plants in the Al-Ahsa oasis during 2018/2019.

Botanical origins		Source		Apiary				
Scientific name	Common name	Nectar	Pollen	1	2	3	4	5
*Brassica napus* L.	Rapeseed	+	+	+	+	+	+	+
*Citrus* spp.	Citrus	+	-	-	+	-	-	+
*Cucurbita pepo* Thunb	Summer squash	+	+	+	+	+	+	+
*Helianthus annuus* L.	Sunflower	+	+	+	+	+	+	+
*Medicago sativa* L.	Alfalfa	+	+	+	+	+	+	+
*Phoenix dactylifera* L.	Date palm	-	+	+	+	+	+	+
*Prosopis* spp.	Mesquite	+	-	+	-	-	+	-
*Ziziphus* spp.	Sidr	+	-	+	+	+	+	+

+ and–indicate source and not source, respectively.

### Sampling of bee pollen

Five colonies of the hybrid Carniolan honeybee (*Apis mellifera* L.) of the same strength were selected in each apiary for this purpose. Pollen traps of 25% efficiency were fitted onto hive entrances. Pollen trap contents were harvested twice a week from 21 March 2018 until 20 March 2019. The harvested pollen loads were classified according to the season: spring (March–May), summer (June–August), autumn (September–November), or winter (December–February).

#### Protein and amino acids preparation and analysis

The nitrogen content was determined in a sample of 0.07 g of bee pollen using the micro-Kjeldahl method. The crude protein was calculated by using a factor of 5.60 for converting nitrogen into crude protein [31]. The method of Szczêsna [27] was used to determine the amino acid profile in bee pollen samples. An LC3000 automatic amino acid analyzer (Eppendorf-Biotronik, Germany) was used for the quantitative and qualitative analyses of the amino acids using ion-exchange chromatography. A sample of 25 mg DM of bee pollen was transferred to a hydrolysis tube containing 10 ml of 6 N HCL. The samples were treated with performic acid to avoid the decomposition of sulfur-containing amino acids [32]. The hydrolysis tube was sealed under vacuum, heated in an oven at 110°C for 24 hrs, and then cooled to room temperature. After hydrolysis, the solution was evaporated, and then dissolved in 1 ml distilled water. The contents were filtered through Whatman No. 1 filter paper to remove visible sediments. The combined filtrate and wash were diluted to the volume of 25 mL in a volumetric flask. Five ml of the filtrate was transferred to a 50 mL beaker. Dry residues were dissolved in 1 mL of lithium citrate buffer (pH 2.2). Twenty μL of the solution was loaded onto the cation exchange column, and then four lithium citrate buffers with pH 2.2, 2.8, 3.3 and 3.7 were successively applied to the column at a flow rate 0.2 mL/min. The ninhydrin flow rate was 0.2 mL/min and the pressure of the reagent was 150 bar. The pressure of buffer was from 0–50 bar and 130°C reaction temperature. The quantitative analysis was performed by comparing the corresponded peak area to those of amino acids.

The article "Effect of harvest season on the nutritional value of bee pollen protein" was retracted in 2022. Reasons: compromised peer review; a conflict of interest; concerns about the authorship.

### Determine the value of bee pollen protein

The chemical score (CS) and EAA index (EAAI) were used to determine the value of bee pollen protein. The EAAI was calculated based on the amino acids in bee pollen and chicken eggs using the equation of [33].

$$\mathrm{EAAI}=\sqrt[{N}]{\frac{\mathrm{Leu}.P\times \ldots \times \mathrm{Met}.P\times }{\mathrm{Leu}.E\times \ldots \times \mathrm{Met}.E}}$$

where (N) indicates the number of EAAs, (P) indicates bee pollen protein, and (E) indicates egg protein [34] as a standard protein.

The equation of Mitchell and Block [35] was used to calculate the CS for the EAAs.

$$\mathrm{CS}=\frac{\mathrm{AAP}\times 100}{\mathrm{AAR}}$$

where (P) indicates the EAAs in the bee pollen protein and (R) indicates the EAAs required by honeybees (*A*. *mellifera*) [24] or adult humans [23].

### Statistical analysis

The differences between harvesting seasons were tested by one-way analysis of variance (ANOVA), which indicated significant differences for harvesting seasons. The normality in data was tested by the Shapiro-Wilk normality test, which indicated data were normally distributed. Therefore, the analysis was performed on the original data. The ANOVA was used to assess differences between the seasons investigated via the PROC GLM function in SAS version 9.1 [36]. Duncan's multiple range test [37] was used to compare treatment means.

## Results

Alfalfa (*Medicago sativa* L.), rapeseed (*Brassica napus* L.), summer squash (*Cucurbita pepo* Thunb), date palm, (*Phoenix dactylifera* L.), and sunflower (*Helianthus annuus* L.) were recorded as the major pollen floral resources in all experimental apiaries. Sidr (*Ziziphus* spp.), Alfalfa, rapeseed, summer squash, and sunflower were recorded as the major nectar floral resources in all experimental apiaries. Citrus (*Citrus* spp.) and mesquite (*Prosopis* spp.) were recorded as major nectar floral resources in apiary 2 & 5, and 1 & 4, respectively (Table 1).

Bee pollen collected during the different seasons showed significant (P < 0.01) variations in protein content and amino acids contents (Table 2). The highest values of protein (20.16 g/100 g DM) and total amino acids (13.04 g/100 g DM) were obtained from bee pollen collected during the spring season. The highest values of total EAAs (5.69 g/100 g DM) and total EAA percentage (43.84%) were obtained from bee pollen collected during the winter season. Bee pollen collected during autumn had the lowest values of amino acids. The values of protein EAAI could be arranged as follows: autumn (62.36%) > summer (60.43%) > winter (59.64%) > spring (58.79%) (Table 3).

The article "Effect of harvest season on the nutritional value of bee pollen protein" was retracted in 2022. Reasons: compromised peer review; a conflict of interest; concerns about the authorship.

**Table 2:** Analysis of variance of protein and amino acids contents of bee pollen.

Variable	SS	MS	F value	P value
Protein	16.99	5.66	292.33	< 0.0001
TAAs	1.15	0.38	80.87	< 0.0001
TEAAs	0.70	0.23	74.80	< 0.0001
TEAAs%	10.01	3.34	282.14	< 0.0001
EAAI	43.77	14.59	467.48	< 0.0001
Leucine	18.65	4.66	152.89	< 0.0001
Valine	5.67	1.42	644.02	< 0.0001
Lysine	5.92	1.48	21.00	< 0.0001
Isoleucine	11.12	2.78	2172.70	< 0.0001
Histidine	25.88	6.47	4256.88	< 0.0001
Threonine	2.48	0.62	721.12	< 0.0001
Arginine	3.85	0.96	280.09	< 0.0001
Phenylalanine	7.65	1.91	1951.78	< 0.0001
Tryptophan	5.45	1.46	1621.66	< 0.0001
Methionine	0.25	0.06	783.00	< 0.0001
Glycine	8.32	12.08	180.98	< 0.0001
Glutamic acid	17.15	4.29	213.56	< 0.0001
Aspartic acid	10.39	2.60	98.30	< 0.0001
Alanine	8.31	2.08	34.29	< 0.0001
Serine	6.58	1.65	931.23	< 0.0001
Tyrosine	5.03	1.26	1521.66	< 0.0001
Cysteine	6.45	1.26	1421.66	< 0.0001
Proline	0.26	0.07	1307.46	< 0.0001

Source of variation = seasons, degree of freedom = 5, SS = sum of squares, MS = mean squares.

TAAS = Total amino acids, TEAAS = Total essential amino acids, EAAI = Essential amino acid index.

**Table 3:** Crude protein, total amino acid and essential amino acid composition of bee pollen.

Season	Protein (g/100 g DM)	TAA* (g/100 g DM)	TEA** (g/100 g DM)	TEA%	EAAI*** (%)
Spring	20.16 ± 0.16^a^	13.04 ± 0.10^a^	5.62 ± 0.06^a^	43.10 ± 0.18^b^	58.79
Summer	19.27 ± 0.14^b^	12.77 ± 0.09^b^	5.44 ± 0.02^b^	42.60 ± 0.21^c^	60.43
Autumn	18.02 ± 0.18^c^	12.46 ± 0.12^c^	5.23 ± 0.03 ^c^	41.97 ± 0.16^d^	62.56
Winter	20.14 ± 0.15^a^	12.98 ± 0.13^a^	5.69 ± 0.03 ^a^	43.84 ± 0.22^a^	59.64
Average	19.40	12.81	5.49	42.86	60.36

Values are the mean ± standard deviation. Means of each column followed by a different letter are significantly different at the 0.01 level.

*–Total amino acids

**–Total essential amino acids.

***–Essential amino acid index (calculated for the 10 essential amino acids).

Ten EAAs and 8 non-EAAs were found in bee pollen collected during all four seasons. The highest contents of leucine (12.85 mg/g), valine (10.26 mg/g), isoleucine (6.50 mg/g), and threonine (4.58 mg/g) were obtained from bee pollen collected during spring. The highest values of lysine (9.66 mg/g), arginine (4.83 mg/g), phenylalanine (3. 24 mg/g), and tryptophan (1.09 mg/g) were obtained from bee pollen collected during winter. Bee pollen collected during autumn showed the highest contents of histidine (6.19 mg/g) and methionine (0.57 mg/g). The highest contents (mg/g DM) of glutamic acid (16.96 mg) and glycine (16.74 mg) were obtained from spring bee pollen, and those of aspartic acid (16.40 mg), alanine (12.65 mg), and proline (0.63 mg) were from summer bee pollen. The highest levels of tyrosine (2.05 mg) and cysteine (1.68 mg) were found in bee pollen collected during the winter season (Table 4).

The article "Effect of harvest season on the nutritional value of bee pollen protein" was retracted in 2022. Reasons: compromised peer review; a conflict of interest; concerns about the authorship.

**Table 4:** Amino acids composition (mg/g DM) of bee pollen.

Amino acid	Spring	Summer	Autumn	Winter	Average
**Essential amino acids**					
Leucine	12.85 ± 0.10^a^	11.94 ± 0.10^b^	10.88 ± 0.10^c^	12.62 ± 0.10^a^	12.07
Valine	10.26 ± 0.11^a^	9.82 ± 0.10^ab^	8.86 ± 0.10^c^	9.98 ± 0.10^a^	9.73
Lysine	8.53 ± 0.06^b^	8.26 ± 0.08^c^	8.38 ± 0.10^c^	9.66 ± 0.08^a^	8.71
Isoleucine	6.30 ± 0.10^a^	6.03 ± 0.10^b^	5.33 ± 0.10^c^	6.05 ± 0.10^b^	5.93
Histidine	4.52 ± 0.03^c^	5.17 ± 0.02^b^	6.19 ± 0.01^a^	4.35 ± 0.02^c^	5.06
Threonine	4.58 ± 0.02^a^	4.57 ± 0.02^a^	4.47 ± 0.01^b^	4.58 ± 0.01^a^	4.55
Arginine	4.39 ± 0.01^b^	4.23 ± 0.01^c^	4.28 ± 0.02^c^	4.83 ± 0.02^a^	4.43
Phenylalanine	3.19 ± 0.02^a^	2.90 ± 0.01^b^	2.51 ± 0.01^c^	3.24 ± 0.01^a^	2.96
Tryptophan	1.06 ± 0.01^a^	0.96 ± 0.01^b^	0.82 ± 0.01^c^	1.09 ± 0.01^a^	0.98
Methionine	0.50 ± 0.01^b^	0.52 ± 0.01^b^	0.57 ± 0.01^a^	0.47 ± 0.01^c^	0.52
**Nonessential amino acids**					
Glycine	16.74 ± 0.12^a^	16.60 ± 0.08^b^	16.52 ± 0.12^c^	16.62 ± 0.09^b^	16.62
Glutamic acid	16.96 ± 0.14^a^	15.83 ± 0.14^b^	15.45 ± 0.13^c^	16.93 ± 0.14^a^	16.29
Aspartic acid	16.21 ± 0.15^b^	16.40 ± 0.12^a^	16.25 ± 0.14^b^	15.63 ± 0.11^c^	16.12
Alanine	12.56 ± 0.11^c^	12.65 ± 0.09^a^	12.61 ± 0.12^b^	12.23 ± 0.10^d^	12.51
Serine	7.65 ± 0.06^c^	7.93 ± 0.04^b^	8.12 ± 0.08^a^	7.34 ± 0.03^d^	7.76
Tyrosine	1.95 ± 0.02^a^	1.81 ± 0.01^b^	1.57 ± 0.01^c^	2.05 ± 0.01^a^	1.85
Cysteine	1.57 ± 0.01^a^	1.43 ± 0.02^b^	1.21 ± 0.01^c^	1.68 ± 0.02^a^	1.47
Proline	0.58 ± 0.01^a^	0.63 ± 0.01^a^	0.59 ± 0.01^a^	0.48 ± 0.01^b^	0.57

Values are the mean ± standard deviation. Means of each row followed by a different letter are significantly different at the 0.01 level.

Leucine, valine, lysine, histidine, threonine, and phenylalanine (except in autumn bee pollen) in all tested samples were above the requirements of honeybees, while leucine, valine, histidine, isoleucine (except in autumn bee pollen), lysine (except in spring and summer bee pollen), and threonine (except in winter and spring bee pollen) in all tested samples were above the requirements of adult humans (Table 5). In comparison with the minimal requirements of adult humans and honeybees, the CS values in the bee pollen samples showed that methionine was the 1^st^ limiting amino acid in all tested samples (Tables 6 and 7).

The article "Effect of harvest season on the nutritional value of bee pollen protein" was retracted in 2022. Reasons: compromised peer review; a conflict of interest; concerns about the authorship.

**Table 5:** Amino acids (g/100 g protein) in bee pollen compared to the minimum requirements of honeybees (*Apis mellifera* L.) and adult humans.

Amino acids	Spring	Summer	Autumn	Winter	Minimum requirements	
					A	B
**Essential amino acids**						
Leucine	6.37	6.20	6.04	6.27	4.50	5.90
Valine	5.09	5.10	4.92	4.96	4.00	3.90
Lysine	4.23	4.29	4.65	4.80	3.00	4.50
Isoleucine	3.13	3.13	2.96	3.00	4.00	3.00
Histidine	2.24	2.68	3.44	2.16	1.50	1.50
Threonine	2.27	2.37	2.48	2.27	1.50	2.30
Arginine	2.18	2.20	2.38	2.40	3.00	-
Phenylalanine	1.58	1.50	1.39	1.61	1.50	-
Tryptophan	0.53	0.50	0.46	0.54	1.00	0.60
Methionine	0.23	0.27	0.32	0.23	1.50	1.60
Phenylalanine + Tyrosine	2.55	2.44	2.26	2.63	-	3.80
**Nonessential amino acids**						
Glutamic acid	8.41	8.21	8.57	8.41	-	-
Glycine	8.30	8.61	9.17	8.25	-	-
Aspartic acid	8.40	8.51	9.02	7.76	-	-
Alanine	6.23	6.56	7.00	6.07	-	-
Serine	3.79	4.12	4.51	3.64	-	-
Tyrosine	0.97	0.94	0.87	1.02	-	-
Cysteine	0.78	0.74	0.67	0.83	-	-
Proline	0.29	0.33	0.33	0.24	-	-

A = Minimal levels of essential amino acids required by the honeybee *Apis mellifera* [24].

B = Minimal levels of essential amino acids required by adult humans [23].

**Table 6:** Chemical score of bee pollen compared to the minimum requirements of honeybees (*Apis mellifera* L.).

Amino acid	Spring	Summer	Autumn	Winter	Average
Leucine	141.56	137.78	134.22	139.33	138.22
Valine	127.25	127.50	123.00	124.00	125.44
Lysine	141.00	143.00	155.00	160.00	149.75
Isoleucine	78.25	78.25	74.00	75.00	76.38
Histidine	149.33	178.67	229.33	144.00	175.33
Threonine	151.33	158.00	165.33	151.33	156.50
Arginine	72.67	73.33	79.33	80.00	76.33
Phenylalanine	105.33	100.00	92.67	107.33	101.33
Tryptophan	53.00	50.00	46.00	54.00	50.75
Methionine	15.33*	18.00*	21.33*	15.33*	17.50*
Average	103.51	106.45	112.02	105.03	106.75

* 1^st^ limiting amino acid

** 2^nd^ limiting amino acid.

**Table 7:** Chemical score of bee pollen compared to the minimum requirements of adult humans.

Amino acids	Spring	Summer	Autumn	Winter	Average
Leucine	107.97	105.08	102.37	106.27	105.42
Valine	130.51	130.77	126.15	127.18	128.65
Lysine	94.00	95.33	103.33	106.67	99.833
Isoleucine	104.33	104.33	98.67	100.00	101.83
Histidine	149.33	178.67	229.33	144.00	175.33
Threonine	98.70	103.04	107.83	98.70	102.07
Tryptophan	88.33	83.33	76.67	90.00	84.583
Methionine	14.38*	16.88*	20.00*	14.38*	16.41*
Phenylalanine + Tyrosine	67.11	64.21	59.47	69.21	65.00
Average	105.04	108.10	112.98	105.25	107.84

* 1^st^ limiting amino acid

** 2^nd^ limiting amino acid.

The article "Effect of harvest season on the nutritional value of bee pollen protein" was retracted in 2022. Reasons: compromised peer review; a conflict of interest; concerns about the authorship.

## Discussion

The concentrations of protein and amino acids in the tested bee pollen samples were significantly (P < 0.01) influenced by the harvesting season. These results confirm the findings of Negrao and Orsi [38]. The variations in amino acids present in pollen among the seasons were due to the diversity of the dominant botanical origins during each season [12,18]. Notable variations in protein and amino acid composition were found among collected bee pollen samples of different botanical origins [12,18,39]. According to Taha [11,30] and Taha et al. [18], the main pollen plants in the Al-Ahsa oasis are sunflower, rapeseed, summer squash, alfalfa, and date palm. All of these plants blossomed during spring; alfalfa, summer squash, and sunflower bloomed during summer. Summer squash blossomed during autumn. Rapeseed, date palm, and summer squash blossomed during winter [11,30]. The highest concentrations of protein, total amino acids, and total EAAs in bee pollen collected during the spring and winter seasons were related to the large proportion of pollen collected from date palm and alfalfa. Bee pollen from these resources had a higher content of amino acids than that of bee pollen with other botanical origins [18,27,40]. Moreover, bee pollen collected during autumn had a lower content of amino acids than of that collected during other seasons because it contained a large proportion of pollen collected from summer squash, which has an insufficient content of protein [11] and amino acids [18].

The predominant amino acids in the tested bee pollens were glycine, aspartic acid, glutamic acid, alanine, leucine, valine, lysine, and serine. Relatively similar results were found by Ghosh and Jung [12] and Taha et al. [18]. The contents of the major amino acids in bee pollen ranged from 7.76 mg/g (serine) to 16.62 mg/g (glycine). These results are in agreement with the findings of Taha et al. [18].

Based on the total quantified amino acids, the EAA content ranged from 41.97% (autumn bee pollen) to 43.10% (spring bee pollen). These values were relatively similar to the values obtained by Taha et al. [18] for Saudi bee pollen but lower than the values obtained by Szczêsna [27] for Polish bee pollen. Based on the total EAA content, leucine was the most predominant EAA in bee pollen collected during spring (22.87%), summer (21.95%), autumn (20.81%), and winter (22.19%), with an average of 21.96% of the total quantified EAAs. Valine was the second most prevalent EAA and constituted 18.26% for spring, 18.05% for summer, 16.94% for autumn, and 17.55% for winter bee pollen, with an average of 17.70%. Similarly, relative percentages were obtained for bee pollen collected from Saudi Arabia [18], Poland [27], and South Africa [19]. On the other hand, lysine was recorded as the most prevalent EAA in Polish bee pollen, while leucine was the second most predominant EAA [41].

The article "Effect of harvest season on the nutritional value of bee pollen protein" was retracted in 2022. Reasons: compromised peer review; a conflict of interest; concerns about the authorship.

The values of glycine, glutamic acid, aspartic acid, alanine, leucine, valine, lysine, and serine in the protein were in the range of Saudi bee pollen [18] but higher than the values of bee pollen from South Africa [19]. The concentrations of lysine, histidine, arginine, methionine, isoleucine, threonine, phenylalanine, tyrosine and proline were relatively similar to the values reported by Taha et al. [18] but lower than the values of Nicolson and Human [19]. These differences were related to differences in botanical origin [12,18].

The composition of protein in bee pollen collected during autumn showed higher concentrations (g/100 g protein) of threonine, histidine, methionine, glutamic acid, aspartic acid, alanine, serine and proline than in pollen collected during other seasons. The high values of the previous amino acids resulted from the low level of protein in bee pollens collected during autumn compared to the proportion of protein in bee pollens collected during the spring and winter seasons.

The nutritive value of bee pollen protein for humans depends on the concentrations of EAAs relative to adult human requirements [23]. Based on the minimal levels of EAAs required by adult humans, leucine, valine, isoleucine, and histidine in bee pollen collected during the four seasons; lysine in autumn and winter bee pollen; and threonine in summer and autumn bee pollen exceeded adult human requirements [23]. The concentrations of tryptophan, phenylalanine + tyrosine, and methionine in all tested bee pollens were lower than adult human requirements [23]. Taha et al. [18] reported a shortage of these amino acids. Except for isoleucine, arginine, tryptophan, and methionine, the EAA in the protein of all bee pollen samples exceeded honeybee requirements [24]. Our results confirm earlier results found by Taha et al. [18].

The nutritive value of bee pollen protein was estimated as CS and compared to the minimum requirements of the honeybee. Based on the CS values of bee pollen protein from different samples, all EAAs apart from isoleucine, arginine, tryptophan, and methionine exceeded the minimum requirements of honeybees [24]. Our values were higher than the values of bee pollen collected in Poland [27]. The highest CS values (%) of bee pollen protein were obtained from bee pollen samples harvested during spring for leucine and isoleucine; winter for lysine, arginine, phenylalanine, and tryptophan; and autumn for histidine, threonine, and methionine.

The article "Effect of harvest season on the nutritional value of bee pollen protein" was retracted in 2022. Reasons: compromised peer review; a conflict of interest; concerns about the authorship.

Based on adult human requirements [23], the highest CS values (%) of bee pollen protein were obtained from spring bee pollen for leucine and isoleucine; winter bee pollens for lysine, tryptophan, and phenylalanine + tyrosine; and autumn bee pollens for histidine, threonine, and methionine. The CS values of bee pollen protein were related to their botanical origins [18].

Based on the minimal requirements of honeybees [24], methionine (15.33%, 18.00%, 21.33%, and 15.33% for bee pollen collected during spring, summer, autumn, and winter, respectively) was the 1^st^ limiting amino acid, followed by tryptophan (53.00%, 50.00%, 46.00% and 54.00%). Similar results were found by Taha et al. [18], Nicolson and Human [19], Szczesna [22], and Hassan [40]. Based on adult human requirements [23], methionine (14.38%, 16.88%, 20.00%, and 14.38% for bee pollen collected during spring, summer, autumn, and winter, respectively) was the 1^st^ limiting amino acid, followed by phenylalanine + tyrosine (67.11%, 64.21%, 59.47%, and 69.21%). Our findings are in agreement with those found by Taha et al. [18].

## Conclusion

The contents of bee pollen protein and amino acids are greatly dependent on the harvest season. The highest contents of crude protein, total amino acids, total essential amino acids, leucine, valine, lysine, isoleucine, threonine, arginine, phenylalanine, tryptophan, glycine, glutamic acid, tyrosine, and cysteine were obtained from bee pollens collected in spring and winter. Bee pollens collected during spring (March–May) and winter (December–February) seasons can be considered an EAA source for adult humans and honeybees.
